The article "Early Diagnosis of Tuberculosis Using Deep Learning Approach for IOT Based Healthcare Applications" was published in 2022. Journal: Comput Intell Neurosci.

# Early Diagnosis of Tuberculosis Using Deep Learning Approach for IOT Based Healthcare Applications

**DOI:** 10.1155/2022/3357508

**Published:** 2022-09-28

**Authors:** G. Simi Margarat, G. Hemalatha, Annapurna Mishra, H. Shaheen, K. Maheswari, S. Tamijeselvan, U. Pavan Kumar, V. Banupriya, Alachew Wubie Ferede

**Affiliations:** ^1^Department of Computer Science and Engineering, New Prince Shri Bhavani College of Engineering and Technology, Chennai, Tamil Nādu, India; ^2^Department of ECE, KSRM College of Engineering, Kadapa, Andhra Pradesh, India; ^3^Department of Electronics and Communication Engineering, Silicon Institute of Technology, Bhubaneswar, Odisha, India; ^4^Department of AIML, Hindusthan College of Engineering and Technology, Coimbatore, India; ^5^Department of Computer Science and Engineering, CMR Technical Campus, Kandlakoya, Hyderabad, Telangana, India; ^6^Department of Radiography, Mother Theresa PG and Research Institute of Health Sciences, Puducherry, India; ^7^Department of ECE, RISE Krishna Sai Prakasam Group of Institutions, Ongole, Andhra Pradesh, India; ^8^Department of Computer Science and Business Systems, M. Kumarasamy College of Engineering, Karur, Tamil Nādu, India; ^9^Department of Chemical Engineering, College of Biological and Chemical Engineering, Addis Ababa Science and Technology University, Addis Ababa, Ethiopia

## Abstract

In the modern world, Tuberculosis (TB) is regarded as a serious health issue with a high rate of mortality. TB can be cured completely by early diagnosis. For achieving this, one tool utilized is CXR (Chest X-rays) which is used to screen active TB. An enhanced deep learning (DL) model is implemented for automatic Tuberculosis detection. This work undergoes the phases like preprocessing, segmentation, feature extraction, and optimized classification. Initially, the CXR image is preprocessed and segmented using AFCM (Adaptive Fuzzy C means) clustering. Then, feature extraction and several features are extracted. Finally, these features are given to the DL classifier Deep Belief Network (DBN). To improve the classification accuracy and to optimize the DBN, a metaheuristic optimization Adaptive Monarch butterfly optimization (AMBO) algorithm is used. Here, the Deep Belief Network with Adaptive Monarch butterfly optimization (DBN-AMBO) is used for enhancing the accuracy, reducing the error function, and optimizing weighting parameters. The overall implementation is carried out on the Python platform. The overall performance evaluations of the DBN-AMBO were carried out on MC and SC datasets and compared over the other approaches on the basis of certain metrics.

## 1. Introduction

In this world, TB (Tuberculosis) is regarded as one of the highest threats to humans and it is considered the fifth major cause of death [1]. It is caused due to *Mycobacterium* and it generally affects the lungs. Further, this bacterium can cause other organs like the brain and kidney. There are two types of TB; they are active and latent TB. In active TB, *Mycobacterium* shows symptoms and it is spread easily; whereas the latent TB, the bacterium stays in the body and does not show any symptoms. Nearly one-fourth of the population has latent TB. During, inhalation, this bacterium is transferred via air from person to person. When proper treatment is given, TB can be cured and prevented using antimicrobial drugs [2]. Based on the 2020 annual report of WHO (World Health Organization) about 11 million people are tested as TB positive. The countries like China, Indonesia, and India are seriously affected due to TB. In addition to this, HIV-affected people died because of TB. Early detection of TB can overcome the advanced explosion of the disease [3]. WHO suggests rapid fundamental tests for TB patients? Hence, automatic CAD (Computer Aided Diagnosis) tools are used for the efficient treatment of TB.

Due to the advancement of computer vision approaches and the advancement of digital techniques several CAD techniques are used recently. With this advancement, TB can be detected quickly and overcome further transmission when it is determined early. CAD has the ability to speed up a mass screening in TB-spreading areas. Traditional examination of chest radiograph technique requires a high professional, is time-consuming, and leads to error. Imaging modalities such as CXR (Chest X-rays) and CT (computed tomography) are generally used to detect and screen for TB. However, the modality CT is not must use due to its cost and high radiation dosage Chest X-rays are mainly used for detecting and diagnosing TB. CXR is a fast, low cost and better tool for early diagnosis [4]. The existing research works on Machine learning (ML) and deep learning (DL) models. ML models are based on hand-crafted features and a DL model does not depend on hand-crafted features. Some of the ML classifiers used in the existing research work are EBT (ensemble baggage tree) [5], RF (Random Forest), [6], and SVM (Support Vector Machine) [7]. Certain research works attained excellent results in DL models. This enables DL as an effective model for medical analysis. Particularly, the DL model CNN (Convolutional Neural Network) has shown better results in TB classification [8–11].

The major contributions of the proposed work are as follows:

- Introduces a fully automated optimized deep learning model for TB segmentation and classification
- Segmentation is carried out by adaptive fuzzy *c* means (AFCM) clustering and features like texture and shape features are extracted
- For improving the accuracy, optimizing weighting parameters, and reducing the error function, a Deep Belief network (DBN) with Adaptive Monarch butterfly optimization (AMBO) is used

The rest of the research article is sorted as Section 2 depicts recent related works based on TB detection; Section 3 explains the developed TB classification model; Section 4 gives the discussion of evaluated results and the entire work is concluded in Section 5.

## 2. Related Works

Some of the recent related works based on TB classification are listed as follows.

Rahman et al. [12] presented a TL (Transfer Learning) with deep CNN for the automatic detection of TB using chest radiographs. The robustness of several CNN approaches was implemented for TB classification. Among the nine models, Chex Net attained better results. The results were evaluated with and without segmentation. It was proved that the classifier with segmentation obtained better outcomes. Win et al. [13] used hybridized feature learning model to screen TB automatically. DeepLabv3 was used for lung segmentation. Then, the optimization PSO (Particle swarm Optimization) was used for selecting features and given as input to optimized SVM. This classifier was used to classify normal and TB. Sahlol et al. [14] used CNN with AEO (Artificial Ecosystem Optimization) for TB detection. Initially, the input image was segmented using MobileNet and, feature selection was carried out by AEO. By this optimization 50,000 features were reduced to 19 and 29 features and classified as TB and Non-TB images.

Pavani et al. [15] presented a new automated model for quick detection of pulmonary TB. At first, preprocessing was carried out and Chan-Vese active contour was used for segmenting the images. Several features were extracted and the pertinent feature was taken for classification by the NB classifier. Rahman et al. [16] integrated DL, a pretrained model, and XGBoost classifier to facilitate the quick diagnosis of TB. The major aim of this research work is to enhance recall and specificity of the classification of TB, furthermore, it minimized the training time in classification. Ayaz et al. [17] used a new TB detection model that integrated hand-crafted features with CNN via an ensemble model. Initially, the images were normalized and given to the feature extractor. GF and pretrained models were used to extract hand-crafted and deep features. Two benchmark datasets were used to obtain better ROC results. Dasanayaka and Dissanayake [18] used several CNN models for automatic TB detection using preprocessing and augmentation approaches. The parameters of the DL models were optimized using a genetic algorithm. Finally, this model attained a detection accuracy of 97.1%. Even though these approaches obtained better results, there were some challenges accompanied by these approaches. Optimization techniques used in these approaches suffered from local optima and the error rate was higher. Hence, there is a robust model is essential for TB detection. Among the top 10 infectious disease-related causes of death, *tuberculosis* (TB) is listed. In this study, convolutional neural networks are used to compare the effectiveness of two approaches for detecting pulmonary *tuberculosis* from patient chest X-ray pictures (CNN). The combination of different picture preparation techniques that produces the highest accuracy is examined. In addition, a hybrid strategy combining the first statistical computer-aided detection method with neural networks was also researched. On the basis of 394 abnormal photos and 406 abnormal images, simulations have been run. The simulations demonstrate that a clipped region of interest combined with contrast augmentation produces superior outcomes. Even better outcomes are obtained when the photos are further enhanced using the hybrid technique [19–28].

## 3. Proposed Methodology

Recently TB classification is carried out by CXR images. The major processes involved in classification are explained in this section. The datasets like Shenzhen China (SC) and Montgomery Country (MC) are used for the process. Initially, the image is resized and noise is removed using the WF filter. Then, the image is segmented using a clustering technique called AFCM. Then, GF, shape, texture, and HoG features are extracted. Finally, a DL model DBN-AMBO is used to classify the image as normal and TB.  Figure 1 delineates the framework of the proposed TB classification model.

### 3.1. Preprocessing

It is an initial phase in image processing. This process is used for removing noise and eliminating unnecessary information. Initially, the input images are resized to 512 × 512 pixels, and this resized image is used for further processing. Then, wiener filtering (WF) is used for removing the noise in a resized image. This filter eliminated an additive noise and removes blurriness at the same time. WF is optimal on the basis of MSE (mean square error). WF is a linear representation of a primary image. WF in Fourier transform (FT) is represented as follows [3]:

(1) $$\begin{array}{c} WF\left(f_{a},f_{b}\right)=\frac{G\left(f_{a},f_{b}\right)T_{zz}\left(f_{a},f_{b}\right)}{{\left|\left(G\;\left(f_{a},f_{b}\right)\right)\right|}^{2}T_{zz}\left(f_{a},f_{b}\right)+T_{mm}\left(f_{a},f_{b}\right)}\text{,} \end{array}$$

where *G*(*f*_*a*_, *f*_*b*_)is blur filter,*T*_*zz*_(*f*_*a*_, *f*_*b*_)is a power spectrum of an image and *T*_*mm*_(*f*_*a*_, *f*_*b*_)is an additive noise.

### 3.2. Segmentation

The preprocessed image is segmented using AFCM. The dataset of *m* samples are *V*={*v*_1_, *v*_2_....*v*_*m*_} and it is partitioned into *c*_*j*_clusters. The objective solution of FCM is [7]

(2) $$\begin{array}{c} K_{n}\left(U,V\right)=\overset{c_{j}}{\underset{l=1}{\sum }}\overset{m}{\underset{p=1}{\sum }}{\left(u_{lp}\right)}^{m}\left(d_{lp}|{}^{2}\right)\text{,} \end{array}$$

where *u*_*lp*_and *d*_*lp*_are the membership degree matrix and Euclidean distance of *l*^*th*^sample and *p*^*th*^centre of cluster. *d*_*lp*_=‖*y*_*l*_ − *v*_*p*_‖The membership degree matrix should satisfy the following conditions:

(3) $$\begin{array}{c} \left\{\sum_{l=1}^{c_{j}}u_{lp}=1,\;l=1,2,....m\right.,\\ 0\leq u_{lp}\leq 1,\;l=1,2,....m,p=1,2....c_{j},\\ 0<u_{lp}<1,\;p=1,2....c_{j}. \end{array}$$

According to Lagrange multiplier, *U*and *V* are computed using the following expression [5]:

(4) $$\begin{array}{c} u_{lp}=\frac{1}{{\sum_{l=1}^{c_{j}}\left(d_{lp}/d_{jp}\right)}^{2/n-1}},v_{p}=\frac{\overset{m}{\underset{p=1}{\sum }}{\left(u_{lp}\right)}^{n}y_{p}}{\overset{m}{\underset{p=1}{\sum }}{\left(u_{lp}\right)}^{n}}\text{.} \end{array}$$

However, the normal FCM has the following limitations it needs an initial matrix of membership and the number of clusters to be declared theoretically. It is largely sensitive to the matrix of membership and number of clusters, therefore FCM generates unstable outcomes. In AFCM, sample density *ρ*_*j*_and density rate *γ*are initialized. The parameter *γ*is utilized for adjusting the potential cluster of centres. In this, *ρ*_*j*_is defined as follows:

(5) $$\begin{array}{c} \rho_{j}=\chi \left(D_{lp}-D_{bo}\right)\text{,} \end{array}$$

where $\chi \left(y\right)=\left\{\begin{array}{c} 1wheny<0\\ 0elsewhere \end{array}\right.$, *D*_*lp*_ is a Euclidean distance of *l*^*th*^sample and *p*^*th*^centre of cluster and *D*_*co*_ is a break off distance. Hence, by using this clustering the TB images are segmented efficiently.

### 3.3. Feature Extraction

Features are used to represent the images in scalar or vector form. Classifiers can not verify an image directly rather than different features like texture and shape features are given as input to the network. In this work, feature extraction is carried out using GF, shape features, and HOG. The explanation about every technique is explained in the following section.

#### 3.3.1. Gaussian Function (GF)

2D GF is utilized for defining the Gaussian function in *G*_*f*_(*a*, *b*) spatial coordination domain. Let *g*(*x*, *y*)is a FT of *G*_*f*_(*a*, *b*) as frequency component function and it is represented as follows [10]:

(6) $$\begin{array}{c} G_{f}\left(a,b,\theta ,\omega ,\alpha ,\mu \right)=\left(\frac{1}{2\pi \sigma_{a}\sigma_{b}}\right)\exp\;\left\{-\frac{1}{2}\left(\frac{a^{2}}{\sigma^{2}}+\frac{b^{2}}{\sigma^{2}}\right)+2\pi i\mu_{a}\right\}\text{,} \end{array}$$

where *θ* and *ω* are the orientation and frequency of GF. In GF, Gaussian is convoluted in the Gaussian window and FT is managed using *α*, *μ*is GF's centre frequency. Then the FT of *g*(*x*, *y*) is represented as follows:

(7) $$\begin{array}{c} g\left(x,y,\theta ,\omega ,\alpha ,\mu \right)=\exp\;\left\{-\frac{1}{2}\left(\frac{{\left(a-\mu \right)}^{2}}{\sigma_{x}^{2}}+\frac{b^{2}}{\sigma_{y}^{2}}\right)\right\}\text{,} \end{array}$$

where *σ*_*x*_ and *σ*_*y*_are the constant distance from the Gaussian properties. *a*=*a*′ cos *θ*+*b*′ sin *θ*, *b* − *b*′ cos *θ*+*b*′ cos *θ*. According to *θ* value several filters are obtained. *θ* value is varied from 45°for obtaining text features.

#### 3.3.2. Shape Features

The flowing features like perimeter, area, Roundness, Eccentricity, Major and minor axes, Ratio of elongation, Solidity, and Equivalent diameter are extracted [4].

*(1) Perimeter *(*P*)* .* It is a number of pixels in the border of object.

*(2) Area *(*A*)* .* It is a space occupied using object on the surface of plane.

*(3) Roundness *(*R*). It is a computation of how closely an object shape to that of circle and it is given as follows:

(8) $$\begin{array}{c} R=\frac{4\pi \times A}{P^{2}}\text{.} \end{array}$$

*(4) Eccentricity *(*E*)* .* This parameter does not have roundness of the object which scales from 0 to 1.

*(5) Major and minor axes.* These are the imaginary ellipse which limits the object.

*(6) Ratio of elongation *(*R*_*e*_)* .* It is a ratio of lengths of major and minor axes and it is defined as follows:

(9) $$\begin{array}{c} R_{e}=\frac{x}{y}\text{,} \end{array}$$

where *x* and *y*are the lengths of minor and major axes.

*(7) Solidity *(*S*)* .* It is a ratio among (*A*) of binary image and convex hull area. It is expressed as follows:

(10) $$\begin{array}{c} S=\frac{A}{A_{con.\;hell}}\text{.} \end{array}$$

*(8) Equivalent diameter *(*E*_*d*_): It is defined as diameter of the circle with a similar area as an object.

#### 3.3.3. HOG

The descriptor in HOG same as the Scale-invariant feature transform (SIFT) and it is obtained in four stages. They are gradient computation, HOG by cells, contrast normalization, and obtaining HOG descriptors. The features of HOG show the presence of TB in the lungs. Let the gradient in pixel (*a*, *b*) in an image *I*_*j*_ is represented as a mask convolution with an original image.

(11) $$\begin{array}{c} G_{a\left(a,b\right)}=Mask_{a}\times I\left(a,b\right)\text{,}\\ G_{b\left(a,b\right)}=Mask_{b}\times I\left(a,b\right)\text{.} \end{array}$$

The gradient magnitude and direction in every pixel (*a*, *b*)are expressed as follows:

(12) $$\begin{array}{c} G_{\left(a,b\right)}=\sqrt{{\left(G_{a\left(a,b\right)}\right)}^{2}{\left(G_{b\left(a,b\right)}\right)}^{2}}\text{,} \end{array}$$

(13) $$\begin{array}{c} \varphi_{\left(a,b\right)}=\arctan\frac{G_{a\left(a,b\right)}}{G_{b\left(a,b\right)}}\text{.} \end{array}$$

Finally, all the three features are integrated and it is given to the classifier. There are 55 features extracted from these features.

### 3.4. Classification

The extracted features are provided as input to the DL classifier DBN. It has input, hidden, and output layers. There is a deep interconnection between input and hidden neurons. The interconnections among hidden and visible neurons are exclusive and symmetric. Since the output of neurons is stochastic in the Boltzmann network is probabilistic. The output is expressed in Equation (14) and the function of the sigmoid is expressed in the following equation:

(14) $$\begin{array}{c} \overset{⟶}{P_{s}}\left(\xi \right)=\frac{1}{1+\exp\;\left(-\xi /s^{p}\right)}\text{,} \end{array}$$

(15) $$\begin{array}{c} \overset{⟶}{QR}=\left\{\begin{array}{c} 1,\;when1-\overset{⟶}{\;P_{s}}\left(\xi \right),\\ 0,\;when\overset{⟶}{\;P_{s}}\left(\xi \right)\text{.} \end{array}\right. \end{array}$$

The deterministic model of stochastic method [8] is expressed as follows:

(16) $$\begin{array}{c} \lim_{s^{p}⟶0}\overset{⟶}{\;P_{s}}\left(\xi \right)=\lim_{s^{p}⟶0}\frac{1}{1+\exp\;\left(-\xi /s^{p}\right)}=\left\{\begin{array}{c} 0,\;when\xi <0,\\ 1/2,\;when\xi =0\\ 1,\;when\xi >0, \end{array}\right.\text{,} \end{array}$$

where *s*^*p*^ is a pseudotemperature? Figure 2 depicts the structure of DBN, in which the process of feature extraction is carried out by RBM (Restricted Boltzmann machine) and classified by MLP (Multilayer proton). The mathematical modeling which expresses the Boltzmann machine energy to form a binary phase is and it is expressed as follows:

(17) $$\begin{array}{c} \Delta e\left(b_{c}\right)=\underset{m}{\sum }b_{c}u_{m,c}+\varphi_{c}\text{,} \end{array}$$

where *u*_*l*_is weight of every neuron and *φ* is bias.

The energy expression on the basis of integration of hidden (*g*, *h*)and visible neurons are provided in equations (18)–(20).

(18) $$\begin{array}{c} E\left(g,h\right)=\underset{\left(c,m\right)}{\sum }g_{c}\;h_{m}\;u_{m,c}-\underset{c}{\sum }k_{c}g_{c}-\underset{m}{\sum }W_{m}h_{c}\text{,} \end{array}$$

(19) $$\begin{array}{c} \Delta E\left(g_{c},\overset{⟶}{h}\right)=\underset{m}{\sum }g_{c}\;h_{m}+k_{c}\text{,} \end{array}$$

(20) $$\begin{array}{c} \Delta E\left(h_{c},\overset{⟶}{g}\right)=\underset{m}{\sum }g_{c}\;g_{c}+W_{c}\text{,} \end{array}$$

where *g*_*c*_ is binary phase of *c*, *W*_*m*_ is a binary phase of *m*hidden unit, *k*_*c*_and *W*_*c*_are the bias provided to the network. For every pair of hidden and visible vector $\left(\vec{h_{i}},\vec{g}\right)$, possibility provided to RBM is given as follows:

(21) $$\begin{array}{c} C\left(\vec{h_{i}},\vec{g}\right)=\frac{1}{p_{f}}\exp\;-E\left(\vec{g},\vec{h}\right)\text{.} \end{array}$$

This approach utilizes CD (contrastive divergence) and its procedure is: training samples are selected and given to visible neurons. Then, find the possibility of hidden neurons and determine the hidden state. Obtain the weight using

(22) $$\begin{array}{c} \Delta w=\alpha \left(\phi^{+}-\phi^{-}\right)\text{,} \end{array}$$

where *α*is a learning rate, *ϕ*^+^and −*ϕ*^−^ are the positive and negative gradients? Every neuron error in *m*is given as follows:

(23) $$\begin{array}{c} e_{m}^{s}={\vec{N}}_{s}-{\vec{R}}_{s}\text{,} \end{array}$$

where ${\overset{⟶}{N}}_{s}$and ${\overset{⟶}{R}}_{s}$ are the input and output vectors. Although DBN has optimized arrangements for classification, several layers are attained experimentally, which degrades its accuracy. So the output achieved by DBN is hybridized with AMBO for enhancing the efficiency of the system. Figure 2 indicates the classification of TB using DBN-AMBO. In MBO [29], butterflies positioned at land 1 and 2 are known as subpopulation *SP*_1_ and subpopulation *SP*_2_. It is computed on the basis of parameters *s* that are *MS*_1_(*Ceil*(*s* × *MS*)) and *MS*_2_(*MS* − *MS*_1_). The individuals of butterflies in *SP*_1_ is operated by migration parameter. It is represented as follows:

(24) $$\begin{array}{c} z_{k,l}^{t+1}=z_{r1,l}^{t}\text{,} \end{array}$$

where *z*_*r*1,*l*_^*t*^is an *l*^*th*^element of *z*_*r*1_. Random position *r*1is chosen from *SP*_1_. When *r* ≤ *s*, *z*_*k*,*l*_^*t*+1^is produced using Equation (24). When *r* > *s*, *z*_*k*,*l*_^*t*+1^is produced using the following equation:

(25) $$\begin{array}{c} z_{k,l}^{t+1}=z_{r2,l}^{t}\text{,} \end{array}$$

where *z*_*r*2,*l*_^*t*^is an *l*^*th*^element of *z*_*r*2_. Random position *r*2is chosen from *SP*_2_. Overall component in butterfly *m*, when *ran* *d* ≤ *s* is given as follows:

(26) $$\begin{array}{c} z_{m,l}^{t+1}=z_{best,,l}^{t}\text{,} \end{array}$$

where *z*_*m*,*l*_^*t*+1^ is an *l*^*th*^element of *z*_*m*_ at *t*+1. *z*_*best*,,*l*_^*t*^is *l*^*th*^element of best butterfly. When *ran* *d* > *s* is given as follows:

(27) $$\begin{array}{c} z_{m,l}^{t+1}=z_{r3,,l}^{t}\text{,} \end{array}$$

where *z*_*r*3,*l*_^*t*^is an *l*^*th*^element of *z*_*r*3_when *ran* *d* > *ARBt* is further given as follows:

(28) $$\begin{array}{c} z_{m,l}^{t+1}=z_{m,l}^{t+1}+\delta \left(az_{m}-0.5\right)\text{,} \end{array}$$

where *ARB*is adjusting rate of butterfly and *az*_*m*_walking stage of the butterfly and *δ* is a weighting factor. However, this optimization suffered from slow convergence and was trapped by local optima. Hence, the crossover operator is introduced to improve the accuracy and to reduce error. In AMBO new individual *z*_*v*_^*t*+1^is given as follows:

(29) $$\begin{array}{c} z_{v2}^{t+1}=\gamma \times C_{o}+z_{v1}^{t+1}\times \left(1-C_{o}\right)\text{,} \end{array}$$

where *C*_*o*_and *γ*are crossover mutation and reflection coefficient. These two parameters improve the performance of TB detection.

## 4. Results and Discussions

This analysis and validation of the DBN-AMBO are depicted in this section. The overall evaluation is carried out on a system with an Intel Core i5 CPU, 8 GB RAM, and 3.0 GHz speed. The overall evaluation is carried out in PYTHON 3.6 platform. The efficiency of the proposed TB classifier is compared against the traditional approaches like RNN (Recurrent Neural Network), CNN, GAN (Generative Adversarial Networks), and DBN. Furthermore, to test the efficiency of optimization techniques, the proposed model is compared with several optimization techniques.

### 4.1. Dataset Details

Shenzhen China (SC) [30] dataset was obtained by Shenzhen number 3 hospital. It comprises 662 frontal CXR images of TB positive images (335) and TB positive images (327). This dataset has images of all age groups of people and these images are in png format which is 0 for non-TB and 1 for TB images. The resolution changes from 998 × 1130 to 3001 × 3001. Montgomery Country (MC) Dataset of frontal CXR images was given by the Health and Human service department of the USA. It comprises 138 frontal CXR images. Among them, 58 are TB positive images and 80 are TB positive images. These images are in png format and their resolution is 4892 × 4020 [31–33].

### 4.2. Performance Measures

It is essential to implement the performance of classification in the studies of image classification. Otherwise, performance will remain incomplete. There are several performance metrics used for classification. In this work, the metrics like Accuracy (A), Recall ®, specificity (S), FNR (False Negative Rate), Precision (P), and NPV (negative predictive value) are measured. The introduced DBN-AMBO evaluated by True positive (exactly classified as TB) (*T*_*p*_), False positive (wrongly classified as TB) (*F*_*p*_), True negative (exactly classified as normal) (*T*_*n*_), and False negative (count of TB cases missed) (*F*_*n*_).

#### 4.2.1. Accuracy

One parameter for assessing classification models is accuracy. Informally, accuracy is the percentage of accurate predictions made by our model.

(30) $$\begin{array}{c} A=\frac{T_{p}+T_{n}}{T_{p}+T_{n}+F_{p}+F_{n}}\text{.} \end{array}$$

#### 4.2.2. Recall

The recall is determined by dividing the total number of Positive samples by the number of Positive samples that were correctly identified as Positive. The model's capacity to identify positive samples is gauged by the recall. More positive samples are found when the recall is higher.

(31) $$\begin{array}{c} R=\frac{T_{p}}{T_{p}+F_{n}}\text{.} \end{array}$$

#### 4.2.3. Specificity

The percentage of true negatives that the model correctly predicts is known as specificity.

(32) $$\begin{array}{c} S=\frac{T_{n}}{T_{n}+F_{p}}\text{.} \end{array}$$

#### 4.2.4. Precision

Precision, or the degree of a successful prediction made by the model, is one measure of the model's performance. Precision is calculated by dividing the total number of positive predictions by the proportion of genuine positives (i.e., the number of true positives plus the number of false positives).

(33) $$\begin{array}{c} P=\frac{T_{p}}{T_{p}+F_{p}}\text{.} \end{array}$$

In Figure 3 illustrates the qualitative analysis of experimental results of the MC Dataset. It shows the preprocessed, segmented images, and classified images.

Table 1 represents the entire performance of the proposed DBN-AMBO with various DL techniques. The approaches like CNN, RNN, GAN, and DBN are exploited for comparison. It is validated from the table that the proposed DBN-AMBO approach obtained better performance in all performance metrics. Specifically, the value of NPV is found to be very low, hence it is efficiently utilized in TB classification.

In Table 2 indicates the entire performance of the DBN-AMBO with recent optimization techniques on the two datasets. DBN-AMBO is compared over DBN-EPO (Emperor penguin optimization), DBN-BOA (Butterfly optimization Algorithm), and DBN- MBO. The accuracy of DBN-AMBO is 9.2%, 5.2%, and 3.1% superior over DBN-BOA, DBN-EPO, and DBN- MBO, respectively.

The CM (confusion matrix) of two datasets for TB classification is provided in Figure 4. This metric is used for evaluating the classification efficiency of the proposed DBN-AMBO. It is the comparison of predicted and true labels in a classification. In a normal case, both datasets provided better outcomes.

Table 3 illustrates the comparison of the running time of several techniques. It is noted from the table that the computational time of the DBN-AMBO is very less when compared with other techniques. That is proposed that DBN-AMBO takes only 0.426 s to complete the implementation process.

Table 4 represents the comparison of the performance with recently published works. When compared to these models, the proposed DBN-AMBO attained better results. This is due to the optimal weight selection by AMBO. This optimizer reduces the loss function and enhances the accuracy.

## 5. Conclusion

TB is a viral infection disease and many countries are affected due to this disease. Hence, each and every TB-positive case should be cured. In this work, a hybrid model was introduced for TB classification using CXR images. This work undergoes four major phases. Initially, the images were preprocessed and segmented. Then, 55 features were extracted and given as input to the classifier. Finally, TB is classified using DBN-AMBO. The overall evaluations were carried out on MC and SC datasets. When comparing these two datasets, the SC dataset obtained better accuracy of 0.992. It is sure that this methodology will facilitate the radiologist in TB classification. Hence, 99% accuracy was achieved by the proposed work while comparing it to other state-of-the-art approaches. In the future, CXR images can be used for TB-affected people who are affected by COVID-19 and pneumonia.

## Figures and Tables

**Figure 1:** A framework of the proposed TB classification model.

**Figure 2:** Classification using DBN-AMBO.

**Figure 3:** Qualitative analysis: (a) input image, (b) preprocessed image, (c) segmented image, and (d) classification.

**Figure 4:** CM: (a) SC dataset and (b) MC dataset.

**Table 1:** Performance of proposed DBN-AMBO with other classifiers.

Datasets	Performance	RNN	CNN	GAN	DBN	DBN-AMBO
Shenzhen China	Accuracy	0.895	0.792	0.972	0.973	0.992
	Precision	0.893	0.927	0.970	0.981	0.978
	Recall	0.935	0.858	0.932	0.934	0.954
	Specificity	0.961	0.718	0.856	0.961	0.991
	NPV	0.214	0.347	0.175	0.283	0.06
	FNR	0.850	0.923	0.971	0.856	0.998

Montgomery Country	Accuracy	0.983	0.894	0.952	0.915	0.987
	Precision	0.853	0.914	0.906	0.913	0.966
	Recall	0.953	0.884	0.926	0.954	0.989
	Specificity	0.862	0.776	0.871	0.964	0.994
	NPV	0.221	0.343	0.074	0.327	0.02
	FNR	0.852	0.913	0.965	0.931	0.972

**Table 2:** Performance of proposed DBN-AMBO with other classifiers.

Datasets	Performance	DBN-BOA	DBN-EPO	DBN-MBO	DBN-AMBO
Shenzhen China	Accuracy	0.852	0.927	0.931	0.992
	Precision	0.871	0.952	0.967	0.978
	Recall	0.915	0.947	0.924	0.954
	Specificity	0.921	0.871	0.941	0.991
	NPV	0.201	0.165	0.275	0.06
	FNR	0.853	0.961	0.852	0.998

Montgomery Country	Accuracy	0.974	0.922	0.914	0.987
	Precision	0.825	0.905	0.935	0.966
	Recall	0.846	0.928	0.941	0.989
	Specificity	0.862	0.811	0.745	0.994
	NPV	0.141	0.065	0.813	0.02
	FNR	0.882	0.835	0.923	0.972

**Table 3:** Execution time of various approaches

Methods	Computation time (s)
DBN	1.52
GAN	3.242
RNN	2.75
CNN	1.348
DBN-BOA	1.771
DBN-EPO	2.721
DBN-MBO	1.74
DBN-AMBO	**0.426**

**Table 4:** Comparison of the performance with recently published works.

Methods	Accuracy	Recall	Specificity
Pavani et al. [15]	0.955	0.933	0.98
Islam et al. [12]	0.90	0.88	0.92
Santhosh et al. [6]	0.86	0.90	0.80
Rahman et al. [16]	0.964	0.966	—
Proposed (Shenzhen China)	0.992	0.954	0.991
Proposed (Montgomery Country)	**0.987**	**0.989**	**0.994**

## Data Availability

The datasets used and/or analysed during the current study are available from the corresponding author on reasonable request.
